The article "Correlation between Serum Levels of Vitamin A and Vitamin D with Disease Severity in Tic Disorder Children" was retracted in 2023. Reasons: unreliable results or conclusions; concerns about the peer review; concerns about the citations.

# Correlation between Serum Levels of Vitamin A and Vitamin D with Disease Severity in Tic Disorder Children

**DOI:** 10.1155/2022/7121900

**Published:** 2022-05-31

**Authors:** Helin Wang, Yali Yang, Dandan Zhou, Chengjie Bai, Minqiang Shi

**Affiliations:** Department of Pediatric, Linping Hospital of Traditional Chinese Medicine, Hangzhou 311106, China

## Abstract

**Purpose:**

To explore and analyze the correlation between serum vitamins A and D levels and disease severity in children with tic disorder.

**Methods:**

A total of 59 children with tic disorders treated in the Linping Hospital of Traditional Chinese Medicine from April 2018 to May 2021 were selected as the observation group. 55 healthy children with matched age and sex who underwent physical examination were selected as the control group. Children in the observation group were subdivided to the mild group (*n* = 35) and moderate-to-severe group (*n* = 24) according to the Yale comprehensive tic severity scale. Afterwards, they were grouped into the temporary group (*n* = 25), persistent group (*n* = 22), and Tourette's syndrome group (*n* = 12) according to their clinical characteristics and course of disease. The severity and serum vitamins A and D levels were collected and compared, and then, Spearman correlation analysis was performed to analyze the correlation between the severity and serum vitamins A and D levels.

**Results:**

Compared with the control group, the serum vitamin A and D levels in the observation group were lower. Compared with the mild group, the serum vitamins A and D levels were lower in the moderate-to-severe group. Spearman correlation analysis revealed a significant negative correlation between disease severity and serum vitamins A and D levels. Regarding the serum D levels, the temporary group > the persistent group > Tourette's syndrome group. There was no significant difference in serum vitamin A levels among the three groups.

**Conclusion:**

Vitamins A and D deficiency in children is strongly associated with tic disorders, and vitamins A and D demonstrate a negative correlation with the severity of tic disorders. Vitamin D is also linked to the clinical type of tic disorder.

## 1. Introduction

Tic disorder is a neuropsychiatric disease with spontaneous muscle twitching as the main symptom and manifestation, with higher occurrence in children [1]. Although the pathogenesis remains unknown, multiple risk factors such as genetics, nerves, immunity, and environment have been identified [2]. According to the onset age, course of disease, clinical manifestations, and presence of vocal tic, it is categorized to transient tic disorder, persistent movement or tic disorder, and Tourette syndrome [3]. Currently, conventional Western medicine is the mainstay, but it is associated with extravertebral reaction, sedation, nausea, and other side effects [4]. Based on the holistic concept and syndrome differentiation, traditional Chinese medicine therapy shows its advantages in the treatment of tic disorders. The tic disorders are treated as per the theory of ZangFu organs, pathological factors, and the differentiation of qi and blood. In addition, nondrug treatments such as acupuncture and massage therapy have been confirmed to be safe via meridian circulation sites and acupoints, which diversifies treatment choices for patients [5, 6].

In recent years, studies have found that tic disorder may be related to dopaminergic disorder, and vitamin D plays an important role in the normal development and function of the dopaminergic system. As such, it is speculated that tic disorder may be related to vitamin D [7]. Studies have shown that blood levels of vitamin D are positively correlated with nervous system functions such as memory, logical analysis, mood, and balance [8]. The decrease of vitamin D is associated with neurodevelopmental disorders in children and psychopsychological problems in adults and neurodegenerative changes in elderly. To our understanding, depression, Parkinson's syndrome, dementia, Tourette disease, obsessive-compulsive disorder, schizophrenia, autism, and other neurological diseases are related to vitamin D deficiency [9]. Vitamin A participates in the maintenance of T cell-mediated immune response and promotes the production of antibodies via immune cells and the production of some cytokines via T lymphocytes [10]. Vitamin A deficiency impairs the immune function of the body by affecting the expression of retinoic acid receptors in immune cells, and it also serves as a risk factor of tic disorder [11].

However, the correlation between vitamins A and D and tic disorder has yet been scarcely explored. To fill the gap, this study intended to analyze the correlation between serum vitamins A and D levels and the severity of the disease in children with tic disorder, with an aim to gain a clear understanding of the pathogenesis and clinical diagnosis and treatment of the disease.

## 2. Materials and Methods

### 2.1. Study Population and Grouping Methods

A total of 59 children with tic disorders treated in the Linping Hospital of Traditional Chinese Medicine from April 2018 to May 2021 were selected as the observation group. 55 healthy children with matched age and sex who underwent physical examination were selected as the control group. Children in the observation group were subdivided to the mild group (*n* = 35, a score <25) and moderate-to-severe group (*n* = 24, a score of 25–50 as moderate, a score of >50 as severe) according to the Yale comprehensive tic severity scale. Afterwards, they were grouped into the temporary group (*n* = 25), persistent group (*n* = 22), and Tourette's syndrome group (*n* = 12) according to their clinical characteristics and course of disease. The children in different subgroups presented comparability. The research was approved by the Ethics Committee of the Linping Hospital of Traditional Chinese Medicine (approved no. 2/97971).

### 2.2. Inclusion and Exclusion Criteria

1. Participants were assessed eligible if they were in line with the diagnosis standard in tic disorders in children [12, 13], could participate in daily life and school activities normally, had not taken healthcare products containing vitamins within 3 months before enrollment of the study, and family members of the children gave informed consent to this trial
2. Participants were assessed ineligible if they had other hereditary, serious organic, nervous system, and mental diseases

### 2.3. Methods

The vitamins A and D in children with tic disorders of different severities and disease types were compared, and then, Spearman correlation analysis was performed to analyze the relationship between the severity and serum vitamins A and D levels. The measurement method of serum vitamins A and D levels: 3 ml of fasting venous blood was extracted from children in different groups, placed in an ordinary biochemical tube, stored in the dark, and determined using high performance liquid chromatography in strict accordance with the instructions.

### 2.4. Statistical Analysis

All data analyses were performed with the SPSS 22.0 statistical software. Enumeration data were expressed as % and compared using the *χ*^2^ test; measurement data were expressed as mean ± standard deviation ($\bar{x}$ ± *s*) and analyzed using one-way ANOVA and multiple post-hoc tests amongst multiple groups followed by the*t*-test between groups. Spearman analysis was used to analyze the correlation between the severity and serum vitamins A and D levels. Statistical significance was assumed at *P* < 0.05.

## 3. Results

### 3.1. Comparison of General Data

There were no significant differences in gender, gestational age, age, birth weight, history of tics, and maternal mode of delivery between the two groups (*P* > 0.05), as given in Table 1.

### 3.2. Comparison of Serum Vitamins A and D Levels

Compared with the control group, the serum vitamins A and D levels in the observation group were significantly lower (*P* < 0.05), as given in Table 2.

### 3.3. Comparison of Serum Vitamins A and D Levels in Different Disease Severities

Compared with the mild tic disorder group, the serum vitamins A and D levels were lower in the moderate-to-severe tic disorder group, and the difference was statistically significant (*P* < 0.05), as given in Table 3.

### 3.4. The Correlation between the Severity and the Levels of Vitamins A and D

Spearman correlation analysis revealed a significant negative correlation between disease severity and serum vitamins A and D levels (*r* = −0.310, *P* < 0.05; *r* = −0.298, *P* < 0.05).

### 3.5. Comparison of Serum Vitamins A and D Levels in Different Clinical Types

Regarding the serum D levels, the temporary tic disorder group > the persistent movement or tic disorder group > Tourette's syndrome group (*P* < 0.05). There was no significant difference in serum vitamin A levels among the three groups (*P* > 0.05), as given in Table 4.

## 4. Discussion

Tic disorder is a genetic heterogeneous disease with complex genetic basis. Intrauterine and extrauterine environmental factors may alter the expression of the genetic phenotype of the disease [14]. As previously noted, immune activation abnormalities and inflammation are strongly linked to human health [15]. Afterwards, the correlation between vitamins A and D and tic disorder has captured extensive attention. Vitamin A is considered to be an essential vitamin for the human body with a variety of biochemical functions, while vitamin A deficiency is a common micronutrient deficiency worldwide. Statistics show that the prevalence of vitamin A deficiency of children is 0.15–4% in China, and vitamin A deficiency is a contributing factor of children's respiratory tract, weakened immunity, neurological dysfunction, and digestive tract dysfunction [16].

In this study, we found that the serum vitamins A and D levels in the observation group were lower than those in the control group, and the moderate-to-severe group was lower than the mild group in serum vitamins A and D levels. Spearman correlation analysis reported a negative correlation between disease severity and serum vitamins A and D levels. Predictably, the more severe the vitamin A and D deficiencies, the more severe the tic disorders. Previously, some experts have analyzed the relationship between vitamin A and its derivatives on the development and function of the nervous system and found that vitamin A can play an important role in the development of the central nervous system in the human embryonic period [17]. It relates to the induction of neural differentiation and neural pattern development and has a direct impact on the proliferation of brain neural stem cells, tissue repair, and regeneration [18]. In addition, a prior study shows that vitamin A has a prominent role in the improvement of immune regulation and symptoms of tic disorders. As a fat-soluble steroid that can be derived from diet or exposure to ultraviolet radiation, vitamin D has been found to be essential in the nervous system and is considered to be a critical neuroactive steroid. Evidence reveals that vitamin D deficiency leads to structural and functional developmental disorders of the brain and hinders the normal transmission of neurotransmitters in the brain, resulting in disorders of the brain system [19]. In a previous study, chronic motor or vocal tic disorder (CTD) children and healthy controls were treated with vitamin D supplement for 3 months (300 IU/(kg^*∗*^D), no more than 5000 IU per day), the serum level of 25 (OH) D was significantly increased in CTD children, and the tic symptoms were significantly improved, which proves that supplementation of vitamin D can be an effective method to improve the symptoms of CTD children [20]. In addition, we found that regarding the serum D levels, the temporary group > the persistent group > Tourette's syndrome group, whereas there was no significant difference in serum vitamin A levels among the three groups. The possible explanation is that the reduction of vitamin D levels has a direct or indirect adverse impact on the development and function of the entire brain, thereby aggravating clinical symptoms and manifestations, which is largely in line with previous research [21, 22].

However, there are few clinical and experimental studies on vitamin D and tic disorders, the direct mechanism of vitamin D deficiency leading to tic disorders is not clear, and the conclusions are not completely consistent. Also, there is no clear reference standard for the dosage and treatment course of vitamin D supplementation intervention in tic disorders, which are all problems to be solved urgently in the future.

## 5. Conclusion

Vitamins A and D deficiency in serum in children is strongly associated with tic disorders, and vitamins A and D demonstrate a negative correlation with the severity of tic disorders. Vitamin D is also connected with the clinical type of tic disorder. Although our study leads the way in examining the association between vitamins A and D and tic disorders, two limitations merit attention. First, the sample size was small. Second, we failed to intervene the children with vitamins A and D to observe the prognosis. Hence, future studies with larger sample size and interventions are warranted.

## Figures and Tables

**Table 1:** Baseline data.

Groups	Control group	Observation group	*t*/*χ*^2^	*P*
*n*	55	59		
Gender (male/female)	35/20	36/23	0.009	0.924
Gestational age (weeks)	39.25 ± 1.24	39.11 ± 1.33	0.582	0.562
Age (years)	7.25 ± 2.11	7.30 ± 2.08	0.127	0.899
Birth weight (kg)	3.39 ± 0.45	3.41 ± 0.42	0.245	0.807
Family history of tics (yes/no)	5/50	8/51	0.207	0.649

**Table 2:** Comparison of the levels of vitamins A and D in serum of the two groups.

Groups	*n*	Vitamin A (mg/L)	Vitamin D (*μ*g/L)
Control group	55	0.36 ± 0.08	26.69 ± 7.52
Observation group	59	0.32 ± 0.07	23.25 ± 8.20
*t*		2.833	2.336
*P*		0.006	0.021

**Table 3:** Comparison of vitamins A and D levels in serum of different disease severities.

Groups	*n*	Vitamin A (mg/L)	Vitamin D (*μ*g/L)
Mild group	35	0.35 ± 0.06	24.69 ± 7.11
Moderate-to-severe group	24	0.26 ± 0.04	21.02 ± 6.25
*t*		6.912	2.094
*P*		<0.001	0.04100.36

**Table 4:** Comparison of vitamins A and D levels in serum of different clinical types.

Groups	*n*	Vitamin A (mg/L)	Vitamin D (*μ*g/L)
Temporary group	25	0.31 ± 0.05	24.16 ± 6.87
Persistent group	22	0.32 ± 0.07	22.93 ± 7.11^*∗*^
Tourette's syndrome group	12	0.32 ± 0.08	20.25 ± 7.25^*∗*^^#^
*F*		0.779	12.587
*P*		0.215	<0.001

^*∗*^ *P* < 0.005, compared with the temporary group, ^#^*P* < 0.005, compared with the persistent group.

## Data Availability

The datasets used during the present study are available from the corresponding author upon request.

## References

[1] Deeb W., Malaty I. A., Mathews C. A. (2019). Tourette disorder and other tic disorders. *Handbook of Clinical Neurology*.

[2] Fernandez T. V., State M. W., Pittenger C. (2018). Tourette disorder and other tic disorders. *Handbook of Clinical Neurology*.

[3] McGuire J. F., Piacentini J., Storch E. A. (2021). Defining tic severity and tic impairment in Tourette Disorder. *Journal of Psychiatric Research*.

[4] Osland S. T., Steeves T. D., Pringsheim T. (2018). Pharmacological treatment for attention deficit hyperactivity disorder (ADHD) in children with comorbid tic disorders. *Cochrane Database of Systematic Reviews*.

[5] Wang F., Ma Z., Li Y. (2021). The clinical intervention choice for pediatric tic disorder patients from a tertiary children’s hospital in China: a large-scale retrospective study based on electronic medical records. *International Clinical Psychopharmacology*.

[6] Wu M., Xiao G. H., Zhang J. M. (2010). Clinical research into qufeng zhidong recipe used to treat 31 children with tic disorder. *Journal of Traditional Chinese Medicine*.

[7] Bond M., Moll N., Rosello A. (2021). Vitamin D levels in children and adolescents with chronic tic disorders: a multicentre study. *European Child Adolescent Psychiatry*.

[8] Tripkovic L., Lambert H., Hart K. (2012). Comparison of vitamin D2 and vitamin D3 supplementation in raising serum 25-hydroxyvitamin D status: a systematic review and meta-analysis. *The American Journal of Clinical Nutrition*.

[9] Berridge M. J. (2018). Vitamin D deficiency: infertility and neurodevelopmental diseases (attention deficit hyperactivity disorder, autism, and schizophrenia). *American Journal of Physiology-Cell Physiology*.

[10] Ahmad S. M., Haskell M. J., Raqib R., Stephensen C. B. (2009). Vitamin A status is associated with T-cell responses in Bangladeshi men. *British Journal of Nutrition*.

[11] Brilot F., Merheb V., Ding A., Murphy T., Dale R. C. (2011). Antibody binding to neuronal surface in sydenham chorea, but not in PANDAS or tourette syndrome. *Neurology*.

[12] Wen F., Gu Y., Yan J. (2021). Revisiting the structure of the yale global tic severity scale (YGTSS) in a sample of Chinese children with tic disorders. *BMC Psychiatry*.

[13] Tagwerker Gloor F., Walitza S. (2016). Tic disorders and tourette syndrome: current concepts of etiology and treatment in children and adolescents. *Neuropediatrics*.

[14] Sun N., Nasello C., Deng L. (2018). The PNKD gene is associated with tourette disorder or tic disorder in a multiplex family. *Molecular Psychiatry*.

[15] Jones H. F., Han V. X., Patel S. (2021). Maternal autoimmunity and inflammation are associated with childhood tics and obsessive-compulsive disorder: transcriptomic data show common enriched innate immune pathways. *Brain, Behavior, and Immunity*.

[16] Chiu M., Dillon A., Watson S. (2016). Vitamin A deficiency and xerophthalmia in children of a developed country. *Journal of Paediatrics and Child Health*.

[17] Weng W. C., Huang H. L., Wong L. C. (2016). Increased risks of tic disorders in children with epilepsy: a nation-wide population-based case-control study in Taiwan. *Research in Developmental Disabilities*.

[18] Wong L. C., Huang H. L., Weng W. C. (2016). Increased risk of epilepsy in children with Tourette syndrome: a population-based case-control study. *Research in Developmental Disabilities*.

[19] Mora J. R., Iwata M., von Andrian U. H. (2008). Vitamin effects on the immune system: vitamins A and D take centre stage. *Nature Reviews Immunology*.

[20] Li H. H., Xu Z. D., Wang B., Feng J. Y., Dong H. Y., Jia F. Y. (2019). Clinical improvement following vitamin D3 supplementation in children with chronic tic disorders. *Neuropsychiatric Disease and Treatment*.

[21] Eyles D. W., Feron F., Cui X. (2009). Developmental vitamin D deficiency causes abnormal brain development. *Psychoneuroendocrinology*.

[22] Zhu C., Zhang Y., Wang T. (2020). Vitamin D supplementation improves anxiety but not depression symptoms in patients with vitamin D deficiency. *Brain and Behavior*.

